The article "Research on Open Oral English Scoring System Based on Neural Network" was retracted in 2023. Reasons: suspected computer-generated content; unreliable results or conclusions; concerns about the data; concerns about the results or conclusions.

# Research on Open Oral English Scoring System Based on Neural Network

**DOI:** 10.1155/2022/1346543

**Published:** 2022-04-23

**Authors:** Xin Wang

**Affiliations:** Department of Foreign Languages, Shandong Women's University, Jinan, Shandong 250002, China

## Abstract

This study designs and implements a scoring system for open-spoken English using NN technology. The system scores the oral recording from the phonetic level and the text level, respectively, and can comprehensively evaluate its oral level. The system will separately score the spoken speech and the spoken content through different scoring models and add the scoring results as the final score, in which the spoken content is obtained by text transcription of the recording by an external speech recognition engine. An acoustic sensor is adopted to collect pronunciation signals of spoken English. Modern signal processing and automatic pattern recognition technology are used to distinguish the quality of spoken pronunciation. Similar semantic units are marked between acoustic feature sequences, which make use of the parallel algorithm processing mode of multi-computing cores of modern GPU and allow multiple units to independently execute the comparison algorithm at the same time. Experiments show that the model in this study achieves better comprehensive scoring performance. The scoring model is of great significance to the development of educational informatization and intelligence, and it also provides a reference for the construction of intelligent oral scoring system.

## 1. Introduction

With the development trend of global economy, being able to master one or more foreign languages is becoming a skill demand of people based on society [1]. Among them, oral English, as a common tool for daily communication, plays an increasingly important role. In traditional English teaching, teachers focus on reading, writing, and listening comprehension and pay little attention to the training of students' “speaking,” which leads to students' limited speaking ability [2]. With the continuous improvement of educational informatization level, the application of computer-assisted language learning (CALL) system in language teaching has become more extensive. The appearance of CALL provides a good learning environment for oral learners. In the CALL system, the key part that can effectively guide learners to learn spoken English efficiently is the scoring mechanism, which focuses on evaluating learners' pronunciation, giving learners effective feedback, and guiding learners to correct their mispronunciations, that is, training and improving learners' ability to speak English [3]. At present, the assessment of spoken English pronunciation is an important topic for computer-assisted spoken English learning [4]. In the oral English test, teachers need to manually correct the oral recordings of a large number of candidates, which is a repetitive and time-consuming job. Using CALL system to realize automatic correction of spoken recording will reduce the workload of teachers [5]. In recent years, with the improvement of computer speed and speech recognition technology, the use of automatic speech recognition (ASR) technology to evaluate spoken speech has become a research hotspot [6]. At present, the CALL system has successfully realized the automatic correction of oral reading questions. However, automatic correction of open-spoken questions is still the research focus to be broken through.

In language teaching, due to the increasing popularity of English teaching in China, the traditional language teaching methods have been unable to meet people's needs [7, 8]. Oral English, as the preferred tool for people's daily communication, is becoming more and more important, making it the most desirable aspect for Chinese people to improve. When there are enough language teachers, giving spoken English and giving feedback on pronunciation evaluation will be of great help to learners [9]. However, the reality is that English teachers are extremely scarce, and even fewer teachers have the ability to teach spoken English. With the rapid development of computer hardware, the computer's computing power is rapidly improved, which makes it possible to process multimedia information in real time [10]. In this context, CALL, as a method for nonnative English speakers to improve their oral English ability, has attracted extensive attention [11]. To provide useful tutoring feedback and improve scoring efficiency, a computer-based automatic scoring system is needed to evaluate the pronunciation quality, fluency, and specific mistakes that nonnative English speakers are prone to make. At present, it is a common means to use computers to help people practice oral English, but there are still some problems. ① Because fluency features are calculated based on human knowledge, some key representations contained in the original data may be lost. ②Each parameter of the model separately is optimized to make the performance of the model in a suboptimal state. Therefore, it is of great research significance and application value to design and implement an intelligent scoring system for open-spoken English [12]. Therefore, this study attempts to use neural network (NN) algorithm to score open-spoken English and try to solve such problems.

With the rapid development of China's economy and the wide application of information technology, an automatic oral English evaluation system based on computer platform is ready to emerge [13]. This system has the following advantages: it will never feel tired and can concentrate on facing every user [14]. People can use it at any time; for some users who are not confident in their spoken English, it is an excellent choice to improve their spoken English in the virtual environment. To solve the problems encountered by the current spoken English evaluation system, this study proposes an open-spoken English scoring method based on NN, which combines learning feature extraction and scoring model from the original time-domain signal input. Similar semantic units are marked between acoustic feature sequences, which make use of the parallel algorithm processing mode of multi-computing cores of modern GPU and allow multiple units to independently execute the comparison algorithm at the same time, thus realizing that the algorithm can analyze larger data sets in a scalable time frame. Through the experimental evaluation, it is concluded that the algorithm proposed in this study has certain advantages in performance, and the scoring result of the proposed method is more accurate.

## 2. Related Work

Literature [15] puts forward a method of scoring spoken English fluency based on convolutional neural network (CNN), which combines learning feature extraction and scoring model from the original time-domain signal input. Literature [16, 17] proposed a scoring mechanism based on HMM and NN technology to promote the improvement of English self-learning ability. Literature [18] pointed out the existing problems of voice scoring mechanism according to the current development situation and compared the advantages and disadvantages of various voice scoring technologies from both subjective and objective aspects. It is proposed that the scoring should be divided into three parts and the scoring mechanism should be constructed. Literature [19, 20] proposed a spoken English recognition algorithm based on sentence segmentation and dynamic programming method and realized the parallel calculation of the algorithm based on GPU. According to literature [21] based on the Gaussian mixture model and automatic recognition algorithm, a text-independent automatic evaluation system for spoken pronunciation, is constructed. According to literature [22] based on the ALZIE platform, a real and useable evaluation system for spoken English is constructed, which can evaluate spoken English pronunciation with high evaluation accuracy. According to literature [23, 24] based on the related technologies of data fusion and oral English evaluation, a method of using data fusion technology to evaluate oral English is proposed. Literature [25] builds a scoring model of spoken English by introducing the Sugeno fuzzy integral to evaluate linking and confusing sounds. Through experimental statistical data, different fuzzy measures and credibility are constructed, and the randomness of natural language and the instability of ASR system are successfully mapped to the Sugeno integral domain.

Based on the in-depth study of related literature and NN technology, this study designs and implements an open oral English scoring system in detail. A general background model is trained with a large number of speech signals. Based on the general background model, the model and features of target distribution are generated based on maximum a posteriori estimation. Based on the study of features such as continuous reading and confusing sounds, the evaluation results of multiple features are fused into comprehensive evaluation results using data fusion technology. In this study, the model is trained and tested using the oral recordings collected from the scene of the situational English test and the corresponding artificial scoring data. The results show that the system has high accuracy and stability for automatic scoring of spoken English. This system will help learners improve their oral English in an all-round way.

## 3. Methodology

### 3.1. NN

Researchers have applied NN technology to image field and natural language processing field, and these fields have also made breakthrough progress [26]. Among them, NN models commonly used in oral comprehension are text CNN model, LSTM model, and transformer network model. The activation function can introduce nonlinear factors into the network, so that NN can approach various nonlinear curves at will, so that the network has more powerful expression ability [27].

The NN of multilayer perceptron is a unidirectional multilayer network structure. There can be different numbers of neurons in each layer of the network structure, and there is no interconnection between neurons in the same layer. The information transmission between network layers only goes along one direction, that is, from input to output. Among them, the first layer is the input layer, all the middle layers are hidden layers of NN, and the last layer is the output layer [28]. CNN model is a typical spatial depth NN model, which can not only obtain the semantic relations between adjacent words but also extract the local features of the text more accurately. The artificial neuron is the most basic unit in NN, and its design inspiration comes from the information transmission mechanism of biological neuron; that is, after a neuron is stimulated, if the stimulus exceeds a certain threshold, this neuron will be activated and transmit information to other neurons. The input data of NN first enter the input layer, and the processing results of the input layer are sent to the hidden layer, where the activation processing is carried out to feedforward to the final output layer. The activation function of nodes in the hidden layer is usually a nonlinear activation function. The working principle of NN is shown in Figure 1.

Back-propagation neural network (BPNN) is a feedforward neural network with multiple hidden layers, and it is one of the most widely used and successful neural networks. CNN is also a feedforward NN, which is very good at dealing with problems related to computer images. CNN can adaptively learn the spatial characteristics of grid data layer by layer through the local connection between neurons, which has translation invariance, so it is often used to solve the problems of classification and recognition in images. The first two layers are used for image feature extraction and dimension reduction, while the full-connection layer maps the extracted features to the final output layer. Organizing multiple neurons according to the layer structure constitutes a complete NN, and the neurons of adjacent layers in the network are connected with each other. NN has two learning stages: forward and reverse.

### 3.2. Speech Processing Technology

Generally speaking, the basic process of computer automatic speech recognition is as follows: ① the recognition system establishes a search grid according to the given grammar and acoustic model library; ②speech signals are collected, the signals are denoised, and speech features are extracted; and ③ the extracted speech features are processed by the decoder, and the decoder finds the most matching one in the search space as the recognition result according to the input speech features. In other words, ASR can be divided into three parts: feature extraction, model base, and pattern matching [29].

Scoring mechanism is the core technology of oral English learning system, and its main purpose is to automatically judge whether a person's English pronunciation is standard or not by computer [30]. Compared with standard pronunciation, similarities and differences with charts are listed, correct pronunciation with sound or animation is prompted, and pronunciation suggestions with voice or text information are given, so that learners can practice repeatedly to improve their English pronunciation. Therefore, it is of practical significance to evaluate pronunciation effectively to guide learners' oral English learning. Fluency feature extraction calculates features highly related to oral English fluency. Sphinx-4 automatic speech recognition (ASR) three systems are characterized by high modularity. Each module is relatively independent of each other. Changing the implementation mode in one module will not affect the work of other modules, and it is highly portable and configurable. Sphinx-4 system structure is shown in Figure 2.

The phonetic scoring technology is to determine the accuracy of the pronunciation made by the speaker. At present, the spoken English learning system can be divided into two categories according to the phonetic scoring technology used. ① Scoring method based on phonetic feature comparison: to evaluate a speech from a subjective point of view, dynamic time warping technology is generally used. ② Scoring method based on acoustic model: this method is objective, mainly based on hidden Markov model technology. The decoder is the core component of the whole system, which is responsible for the construction of the system search grid and the pattern matching of the input speech features. Sphinx-4 gets the most likely word sequence through the result parser and outputs it as the final recognition result. The system does not require all applications to adopt the field mode. Users can use the output of any processing unit as the input of the system to drive the system to complete the identification process. Therefore, it is not difficult to see that Sphinx-4 has strong configurability.

### 3.3. Design and Implementation of an Open-Spoken English Scoring System

To realize the automatic evaluation of spoken English, the signal analysis method of spoken English pronunciation is used to evaluate the quality and extract the signal features, and the extracted quality features of spoken English pronunciation are adaptively matched. After calling the scoring model module, the trained scoring model is loaded to automatically correct the spoken English data, and the scoring results are saved in Excel file format.

For the scoring model based on BPNN, the data processing module is mainly used to extract features from spoken recording and speech recognition text. In the scoring model, this module is mainly used to convert spoken recording and speech recognition text into numerical vector representation. In addition, the module also provides data cleaning function. An acoustic sensor is adopted to collect pronunciation signals of spoken English. The scoring model is a function that assigns the score *y* to the unknown fluency feature *x*, as shown in the following formula:

(1) $$\begin{array}{c} f\left(x;\theta \right)\mathrm{=y}, \end{array}$$

where *θ* is a set of parameters; *x* is an N-dimensional feature vector; and *y* is a scalar value. Therefore, the features of the scoring model are the input feature *x* and the model parameter *θ*.

The suprasegmental features of speech, also known as prosodic features, mainly include sound intensity, pitch, and length. Pronunciation shows the stress, light tone, and other changes of speech. Pitch shows the tone and intonation of speech, while duration shows the rhythm of speech. Previously, the evaluation of phonetic suprasegmental mainly focused on the evaluation of phonetic length; that is, the speech was scored according to the speech speed or segmental length, but only the rhythm of the speech was evaluated, and the score obtained was one-sided and not accurate enough. The original audio data are segmented for the first time, and the segmentation boundary is defined according to the silence area. The evaluation module of the system mainly evaluates and analyzes the scoring results of the scoring model, including calculating Pearson's correlation coefficient, average score difference, and scoring accuracy of the system between the system scoring and manual scoring. At the same time, the module can also visually analyze the scoring results of different scoring models.

Assuming that the basic scoring unit is phoneme and Γi is the starting time of the ith phoneme, the scoring formula is as follows:

(2) $$\begin{array}{c} l_{i}=\sum_{t=\Gamma_{i}}^{\Gamma_{i}+1-1}\log\left(p\left(s_{t}|s_{t-1}\right)p\left(x_{t}|s_{t}\right)\right), \end{array}$$

where *x*_t_ and *s*_t_ are the observation vector and the state of the model at time *t*, respectively. P(*s*_t_|s_t-1_) is the transition probability. P(*x*_t_|*s*_t_) is the output probability distribution of state st. For each frame corresponding to the ith segment of the phoneme *q*_i_, the frame-based posterior probability P(*q*_i_|*x*_t_) of the phoneme *q*_i_ is calculated as follows:

(3) $$\begin{array}{c} p\left(q_{i}|x_{i}\right)=\frac{p\left(x_{t}|q_{t}\right)p\left(q_{t}\right)}{\sum_{q-1}^{M}p\left(x_{t}|q\right)p\left(q\right)}, \end{array}$$

where p(*x*_t_|q) is the probability density of the current observation, and the sum on the denominator is the total sum of all text-independent phonemes *q* = 1,...,M. Similar to the likelihood log score, the frame-based posterior probability log score is obtained by accumulating all frames in the ith segment:

(4) $$\begin{array}{c} p_{i}=\sum_{t=\Gamma_{i}}^{\Gamma +1-1}\log\left(p\left(q_{i}|x_{i}\right)\right). \end{array}$$

Each evaluation index consists of three scores: accuracy, recall rate, and F value. As shown in the following formula:

(5) $$\begin{array}{c} \text{Precision}=\frac{\left|\mathrm{algorithm}\;\mathrm{identification}\cap \mathrm{standard}\;\mathrm{words}\right|}{\left|\mathrm{algorithm}\;\mathrm{identification}\right|}\\ \text{Recall}=\frac{\left|\mathrm{algorithm}\;\mathrm{identification}\cap \mathrm{standard}\;\mathrm{words}\right|}{\left|\mathrm{standard}\;\mathrm{words}\right|}\\ \mathrm{F-}\text{Score}=\frac{2\times \mathrm{algorithm}\;\mathrm{identification}\times \mathrm{standard}\;\mathrm{words}}{\mathrm{algorithm}\;\mathrm{identification}+\mathrm{standard}\;\mathrm{words}}. \end{array}$$

Nonstandard voices are collected and graded by language experts to form a graded scoring model. For the learner's voice extraction features, the predefined language model and the trained acoustic model are used to force alignment, and the scoring results are obtained through the appropriate scoring mechanism. The accuracy of speech recognition system will directly affect the accuracy of scoring model, so it is very important to choose a suitable speech recognition engine. Word error rate is used to describe the accuracy of speech recognition engine. At first, the system will record the voice input by the user. After the user input is completed, the user input will be recognized by voice, and the result of the recognition will be expanded by grammar. Then, the linking and confusing sounds will be evaluated separately. Finally, the evaluation results of the two will be synthesized and the comprehensive evaluation results will be given.

Multilayer wavelet feature scale transform is used to decompose the features of spoken English pronunciation signals, and it is found that there is a one-to-one mapping relationship between pronunciation quality output independent phase R^N^ and X^N^:

(6) $$\begin{array}{c} p\left(R^{N}=r_{i}\right)=p\left(\begin{array}{c} X^{N}=x_{i}|\left|x_{i}\right|=\left|r_{i}\right|,\text{ angle}\left(x_{i}\right)\\ =\left(\text{angle}\left(r_{i}\right)-\phi_{g}\right)\mathrm{mod}\left(2\pi \right) \end{array}\right). \end{array}$$

When the phase distribution angle (X^N^) of the spoken English pronunciation signal output by noise reduction is uniformly distributed on [0, 2*π*), R^N^ and *φ*_g_ are independent, and it is obtained within the distribution range of the energy set {*P*_1_, *P*_2_,…,*P*_j_}. Take the relationships between the phase information and the phase distribution angle into consideration; formula 6 can be transferred to the following formula:

(7) $$\begin{array}{c} H\left(X^{N}|Z^{N}\right)=H\left(R^{N}|Z^{N}\right)+H\left(\phi_{g}|Z^{N}\right). \end{array}$$

Extracting the wavelet entropy features of spoken English pronunciation signals is as follows:

(8) $$\begin{array}{c} H\left(R^{N}\right)=-\overset{M}{\underset{i=1}{\sum }}p\left(r_{i}\right)\log\left(p\left(r_{i}\right)\right)=-\overset{M}{\underset{i=1}{\sum }}p\left(x_{i}\right)\log\left(p\left(x_{i}\right)\right)=H\left(X^{N}\right), \end{array}$$

where *M* is the number of elements in the symbol set. The adaptive filter coefficient of the spoken English pronunciation signal is as follows: *N*^(1)^=*N*,  *N*^(*j*)^=*N*_0_^(*j* − 1)^,  2 ≤ *j* ≤ *J*. According to the above signal analysis, intelligent speech recognition is performed to improve the automatic evaluation ability of the spoken English pronunciation quality.

To find out the mean and variance at each moment, first a learning sample sequence is selected as the core sample, and then a similar learning data are input to match with the core sample to find the best path function. Intelligent oral scoring refers to the dynamic process from audio input to total score output. The data processing module extracts voice features and text features from clean recording and speech recognition texts, respectively, and inputs these two features into the speech scoring model and the text scoring model, respectively.

## 4. Result Analysis and Discussion

After the stages of speech noise reduction, speech recognition, and data processing, we got the input data of NN scoring model, and combined with the tag data, we can train and test the scoring model accordingly. When training NN, the three kinds of scores in the machine scoring of each nonstandard speech are taken as an input, and the artificial scoring is taken as the expected output, the training times are set, NN is constructed according to the needs, and a required NN is obtained, that is, the scoring mechanism of nonlinear mapping after training. To prove that the features learned by NN algorithm have good discrimination, this study makes a classification experiment on TIMIT database. Random training and test samples are selected, support vector machine is used as classifier, and the classification effect is shown in Figure 3. The data in the figure show that this algorithm is used for feature extraction of speech signals, and the learned features have stronger resolution performance than other algorithms.

The whole system construction needs a lot of hyperparameters; for example, in feature selection, it is necessary to select the feature dimension, the length of each frame speech, and whether there is overlap between frames, and if so, how long the overlap is. Loudness psychology is a measure of human auditory perception, which indicates the intensity of sound energy. We can extract the loudness characteristics of speech and make a loudness curve. First, the speech is mapped from the frequency domain to the perception domain by a certain function. Then, in the loudness domain, the loudness difference between standard speech and test speech is dynamically regularized to obtain the perception score.

The network needs to adapt to these data with different values, so the model becomes difficult to converge. Therefore, it is necessary to standardize the teacher's manual grading data and input characteristic values before training NN. The test method is to count the evaluation results of each sentence in each group and calculate the proportion of each evaluation result and the value of the objective function to determine the performance and stability of the algorithm. Because of the evaluation of continuous reading, it is necessary to compare the recognition result with the sentence processed by continuous reading rules to give an evaluation result. To verify the performance of this algorithm, we select the traditional algorithm, deep learning (DL) algorithm, and this algorithm to carry out comparative experiments of various indexes.  Figure 4 shows the accuracy comparison of the three algorithms.

As can be seen from the figure, compared with the traditional algorithm and DL algorithm, the accuracy of this algorithm is higher. It has a certain accuracy. The comparison of recall rates of the three algorithms is shown in Figure 5.

According to the trend analysis in the figure, the recall rate of our algorithm is the best among the three algorithms, the traditional algorithm is the worst, and the DL algorithm is the best. The comparison of F values of different algorithms is shown in Figure 6.

It can be seen from the analysis that the F value of this algorithm is higher than the other two algorithms in the comparison of F values of different algorithms. Experiments show that the algorithm in this study achieves high matching accuracy on the basis of zero recall rate and F value, which indicates that the matching has good similarity, but there is still a certain gap compared with manual listening and translation. Through the analysis of the experimental evaluation data, it is known that the identification method in this study can find a large number of sentence units while maintaining relatively high matching accuracy.

In this study, the accuracy of scoring results is defined by establishing a maximum value of human-machine scoring error. The main functions of this model are as follows: for a given grammar sentence, according to the existing linking rules, all linking possibilities in the grammar text are marked, all possible linking extensions are generated, and new compound words are added to the dictionary of the system. In particular, in the fluency feature, in the experiment, it is found that the recording with more pauses tends to have a low score. The accuracy of open oral English assessment by different methods is tested, and the comparison results are shown in Figure 7.

Analysis of Figure 7 shows that the accuracy of this method is higher than that of the other two methods. From this, it can be concluded that the open oral English assessment system is accurate and stable. Coverage represents the percentage of complete matching pairs that exist in the grouping set. Grouping rate and type rate evaluate the homogeneity of grouping clusters. The token score compares the subdivision boundary of the word unit with the standard word boundary. The number of boundaries is the number of word unit boundaries identified by the algorithm. Multicore computing is very important. If multicore parallel computing is not possible, the time cost will be very high, and the increase in time cost means that we do not have more energy to test more parameters, which will eventually affect the performance of the whole system.

The index emphasizes that the trade-off between a large number of limited statement units and a small number of statement units can be found accurately. Based on the coverage rate of the recognition method described in this study, the high score closest to manual listening and translation is obtained, which means that this method finds the largest part of a set of repetitive patterns.

This study has done many experiments to improve the performance of the system through the selection of parameters, but with so many parameters, it is almost foreseeable that if the parameters can be selected more reasonably, the performance of the system will be further improved. Using this system to automatically evaluate the pronunciation quality of spoken English has high accuracy, good stability, and good application value.

## 5. Conclusions

NN's hierarchical representation of data using unlabeled data has gained a lot of attention. However, it is one of the greatest challenges of our time for computers to understand complex and high-dimensional audio data. To enable nonnative English speakers to learn spoken English well and score students' spoken English with a unified judgment basis, this study proposes an open scoring method for spoken English based on NN technology. This method comprehensively evaluates different aspects of students' oral English and finally obtains the students' oral English scores.

This study summarizes NN technology and speech scoring technology. There are key and user-defined parameters in the algorithm, and the selection of these parameters determines the quality of the algorithm results. These parameters include feature smoothing window size, quality threshold, and reward and penalty weight. This study defines a set of index system for evaluating algorithm performance. In the experimental part, the performance of the proposed method is evaluated using the existing data sets, the optimal structure is found, and the method is verified. The results show that the machine score using NN is closer to the expert score, and it has certain accuracy and practicability. It is concluded that the proposed method is feasible and an effective means to realize real-time recognition of spoken English. Although the scoring system realized in this study achieves good scoring performance and has certain practicability, it still has some problems. Future work is to further try to improve the efficiency of the proposed algorithm without sacrificing its high accuracy.

## Figures and Tables

**Figure 1:** Working principle of NN.

**Figure 2:** Sphinx-4 system architecture.

**Figure 3:** Comparison of characteristic performance of different algorithms.

**Figure 4:** Accuracy comparison of three algorithms.

**Figure 5:** Comparison of recall rates of three algorithms.

**Figure 6:** Comparison of F values of three algorithms.

**Figure 7:** Comparison of the accuracy of open oral English assessment with different methods.

## Data Availability

All the data are included in this study.

## References

[1] Bartolotti J., Bradley K., Hernandez A. E., Marian V. (2017). Neural signatures of second language learning and control. *Neuropsychologia*.

[2] Ermáková A., Kopivová M. (2018). Corpus-based research of spoken language: the state-of-the-art for Czech and English. *Slovo a Slovesnost*.

[3] Kozo J., Wooten W., Porter H., Gaida E. (2020). The partner relay communication network: sharing information during emergencies with limited English proficient populations. *Health Security*.

[4] Kirkpatrick R. (2016). *English Language Education Policy in Asia. Language Policy*.

[5] Zhang X. (2016). English language education in China: a historical, social and economic perspective. *English Today*.

[6] Paquette-Smith M., Cooper A., Johnson E. K. (2020). Targeted adaptation in infants following live exposure to an accented talker. *Journal of Child Language*.

[7] Levy E. S., Moya‐Galé G., Chang Y. M. (2020). Effects of speech cues in French–speaking children with dysarthria. *International Journal of Language & Communication Disorders*.

[8] Villwock A., Wilkinson E., Piñar P., Morford J. P. (2021). Language development in deaf bilinguals: deaf middle school students co-activate written English and American Sign Language during lexical processing. *Cognition*.

[9] Mpofu N., Maphalala M. C. (2021). English language skills for disciplinary purposes: what practices are used to prepare student teachers?. *South African Journal of Education*.

[10] Sigurjónsdóttir S., Nowenstein I. (2021). Language acquisition in the digital age: L2 English input effects on children’s L1 Icelandic. *Second Language Research*.

[11] Dincer A. (2020). Review of Flipping academic English language learning: experiences from an American university. *Language, Learning and Technology*.

[12] Kambanaros M., Giannikas C. N., Theodorou E. (2020). English foreign language teachers’ awareness of childhood language impairment. *Clinical Linguistics and Phonetics*.

[13] Jain G. (2019). English language competency: need & challenge. *Science, Technology & Human Values*.

[14] Mizrahi R., Creel S. (2019). Preschool[-aged] children’s use of perceptual features to identify spoken languages. *Journal of the Acoustical Society of America*.

[15] Lin L., Liu J., Zhang X., Liang X. (2021). Automatic translation of spoken English based on improved machine learning algorithm. *Journal of Intelligent and Fuzzy Systems*.

[16] Biller M. F., Johnson C. J. (2020). Examining useful spoken language in a minimally verbal child with autism spectrum disorder: a descriptive clinical single-case study. *American Journal of Speech-Language Pathology*.

[17] Nygaard L. C. (2018). Experience, attention, and context in the processing of systematic variation in spoken language. *Journal of the Acoustical Society of America*.

[18] Yakup M. (2018). The acquisition of English stress by Kazakh-Russian bilinguals: the role of dominant language. *Journal of the Acoustical Society of America*.

[19] Do M. N., Lee J. Y., Kim J. R. (2018). Development of level-differentiated flipped learning model for teaching and learning English language in Korean primary school. *Asia Life Sciences*.

[20] Tantucci V., Wang A. (2018). Illocutional concurrences: the case of evaluative speech acts and face-work in spoken Mandarin and American English. *Journal of Pragmatics*.

[21] Raisanen T. (2020). The use of multimodal resources by technical managers and their peers in meetings using English as the business lingua franca. *IEEE Transactions on Professional Communications*.

[22] Yu P., Pan Y., Li C. (2016). User-centred design for Chinese-oriented spoken English learning system. *Computer Assisted Language Learning*.

[23] Pérez-Paredes P., Bueno-Alastuey M. C. (2019). A corpus-driven analysis of certainty stance adverbs: obviously, really and actually in spoken native and learnerEnglish. *Journal of Pragmatics*.

[24] Leuckert S., Rüdiger S. (2020). Non-canonical syntax in an expanding circle variety. *English World-Wide*.

[25] Allan R. (2018). Lexical bundles from one century to the next. *Journal of Historical Pragmatics*.

[26] Winter B., Perlman M., Majid A. (2018). Vision dominates in perceptual language: English sensory vocabulary is optimized for usage. *Cognition*.

[27] Du H., Guan H. (2016). Hindrances to the new teaching goals of College English in China. *English Today*.

[28] Carretero M. (2020). Epistentiality, manner and dialogic contraction: the case of English clearly and Spanish claramente. *Journal of Pragmatics*.

[29] Adokorach M., Isingoma B. (2020). *Homogeneity and Heterogeneity in the Pronunciation of English Among Ugandans: A Preliminary Study*.

[30] Chohan M. N., García M. I. M. (2019). Phonemic comparison of English and punjabi. *Journal of English Linguistics*.

